# Acidic pH promotes nucleus pulposus cell senescence through activating the p38 MAPK pathway

This article has been retracted.

**DOI:** 10.1042/BSR20181451

**Published:** 2018-11-14

**Authors:** Jiabin Fu, Wei Yu, Dianming Jiang

**Affiliations:** 1 Department of Orthopedics, Chongqing Medical University, Chongqing 400016, China; 2 Department of Orthopedics, Inner Mongolia Baogang Hospital, Baotou, Neimenggu 014010, China

**Keywords:** intervertebral disc, nucleus pulposus, pH, p38 MAPK, senescence

## Abstract

Background: Nucleus pulposus (NP) cell senescence is an important cellular feature within the degenerative disc. It is known that a very acidic niche exists in the degenerative disc, which participates in regulating disc cell viability and matrix metabolism. Objective: The present study was aimed to investigate the role and potential signaling transduction pathway of an acidic pH in regulating NP cell senescence. Methods: Rat NP cells were cultured in an acidic pH of 7.2 close to that in a healthy disc (Control group) or in an acidic pH of 6.2 close to that in a severe degenerative disc (Experiment group) for 10 days. Additionally, the experimental NP cells were incubated along with the inhibitor SB203580 to analyze the role of p38 MAPK pathway in this process. Results: Compared with the control NP cells, experimental NP cells showed a suppressed cell proliferation potency, an increased G_0_/G_1_ phase fraction whereas a decreased S-phase fraction and a declined telomerase activity, an up-regulated expression of senescence-related molecules (p16 and p53), and a down-regulated expression of matrix-related moleucles (aggrecan and collagen II). Further analysis showed that inhibition of the p38 MAPK pathway partly reversed effects of acidic pH of 6.2 on the experimental NP cells. Conclusion: The very acidic niche identified in a severe degenerative disc promotes NP cell senescence through regulating the p38 MAPK pathway. The present study provides a new mechanism that drives NP cell senescence during disc degeneration.

## Introduction

Low back pain (LBP) is a leading cause of disability, which affects approximately 85% adults and brings a heavy socioeconomic burden on the public healthcare system [1]. Apart from the unhealthy lifestyle and acute mechanical injury, intervertebral disc degeneration (IDD) is the main contributor to LBP [2]. Currently, treatments for LBP mainly focus on relief of pain symptoms rather than biological regeneration of the degenerative disc or retarding of the pathological progression of disc degeneration [3]. The key bottleneck of this dilemma is lack of well-recognized pathogenesis of disc degeneration.

The intervertebal disc (IVD) consists of three structurally connective parts: peripheral annulus fibrosus (AF), the central gelatinous nucleus pulposus (NP), and the cartilage endplates (CEPs) [4]. The IVD is the largest avascular organ in human body [5]. Essential cell nutrients, such as oxygen, glucose, and animo acids, are mainly supplied to the disc cells by diffusion from the blood vessels at the disc margin or nutrition channels in the CEP [6]. It is estimated that adult human disc NP cells are 7–8 mm from the peripheral nutrient supply [7]. Just because of these reasons, the oxygen within the central disc NP tissue is very low, which leads to an increase in lactate production of NP cells and thus an acidification niche within the NP region [8]. With ageing and disc degeneration, the pathological alterations of CEPs including calcification, lesion, and hypertrophy will further limit nutrients’ diffusion into the central NP and ultimately impede metabolic products flow out of the central NP [9–11]. Hence, the pH value of central NP tissue ranges from 7.2 in a healthy disc to 6.2 in a severe degenerative disc [12].

It has been known that a physiological pH is important to retain normal cell function whereas an extremely low acidic pH induces cell apoptosis and structural changes in extracellular matrix [13]. To date, several studies have demonstrated that an acidic niche can change biological activities of human and/or animal NP cells, including inducing cell apoptosis, inhibiting cell proliferation and promoting matrix catabolism [14–18]. During disc degeneration, cellular senescence is a classical feature within the NP region [19]. Importantly, acidic pH can induce epithelial cellular senescence in reflux esophagitis [20]. However, the effects of acidic pH on NP cell senescence is unclear.

In the present study, we cultured NP cells in different acidic pH environments including an acidic pH of 7.2 close to that in a healthy disc and an acidic pH of 6.2 close to that in a severe degenerative disc. We mainly aimed to investigate effects of acidic pH on NP cell senescence and the involved signaling pathways. NP cell senescence was evaluated by cell proliferation, telomerase activity, cell cycle analysis, and expression of senescence markers.

## Materials and methods

### Ethical statement

All experiments in the present study were approved by the Ethics Committee at Chongqing Medical University [SNY(YU) 2002-0237].

### NP cell collection and culture

Rat lumbar discs (L1–L6) were separated from 25 healthy Sprague–Dawley rats (5 weeks old and 240–260 g weight) within 2 h after killing. Then, the central NP tissues were obtained as described previously [21] and placed in standard DMEM/F12 culture medium (Gibco, U.S.A.). NP cells were isolated by digestion with 0.02% collagenase for 9–12 h at 37°C. Then, the collected NP cell pellets were pre-cultured with DMEM/F12 medium with 10% FBS (BSA, Gibco, U.S.A.). After NP cells grew to 80–90% confluence, they were dismissed by 0.25% trypsin (Gibco, U.S.A.) and re-suspended. In the present study, the passage-two NP cells were used in each assay. The control NP cells (Control group) were cultured in culture medium with an acidic pH of 7.2 whereas the experimental NP cells (Experiment group) were cultured in culture medium with an acidic pH of 6.2 for 10 days in a humid atmosphere (37°C, 21% O_2_ and 5% CO_2_). The pH value of culture medium was adjusted by HCl and NaOH using a pH meter (Meacon Company, China). Additionally, the inhibitor SB203580 was incubated along with the experimental NP cells (Experiment + SB203580 group) to investigate the role of the p38 MAPK pathway in this process.

### Cell proliferation analysis

NP cell proliferation was evaluated by CCK-8 assay and EdU incorporation assay. NP cells were seeded in the six-well plate (2 × 10^3^ cells/well) and incubated for 3 or 7 days in different acidic culture media. Then, one group of NP cells were used to perform the CCK-8 assay according to the manufacturer’s instructions (Beyotime, China). Another group of NP cells were used to measure EdU incorporation ability using a Click-iT EdU microplate assay kit (Invitrogen, U.S.A.). In these two assays, NP cell proliferation potency was expressed as the absorbance at 450 nm wavelength and as the relative fluorescence units (RFUs) detected at an excitation/emission wavelength of 490/585 nm, respectively.

### Cell cycle analysis

The cellular fraction of the G_1_/G_0_, S, and G_2_/M phases after nuclear staining with propidium iodide (PI) was analyzed to detect cell cycle changes. Briefly, after a 10-day acidic culture, NP cells were dismissed by 0.25% trypsin without EDTA. Then, after NP cell pellets were fixed with 75% ethanol for 24 h, they were incubated with RNase A (1 mg/ml) and PI (50 μg/ml, Beyotime, China) for 30 min. Finally, the processed NP cells were subjected to a flow cytometry machine to analyze cell cycle phases (G_0_/G_1_, G_2_/M, S) using the multicycle software (Japan PHENIX Company).

### Telomerase activity detection

Telomerase activity was analyzed by a telomerase (TE) ELISA kit (Mlbio Company, China). Specifically, NP cells were seeded in the 10-cm diameter dish (5.0 × 10^4^ cells/dish) and incubated with different acidic culture medium for 10 days. NP cell pellets were then lysed using the lysis buffer and the supernatant was used to measure the telomerase activity (IU/l) according to the manufacturer’s instructions. A standard curve was developed using the standards provided by the commercial kit. Finally, telomerase activity of samples was calculated according to the absorbance values at 450 nm wavelength and the standard curve.

### Real-time PCR analysis

The mRNA expression of matrix-related molecules (aggrecan and collagen II) and senescence-related molecules (p16 and p53) was assessed by real-time PCR analysis. Briefly, after total RNA sample was collected using the TRIzol solution (Invitrogen, U.S.A.) and then reverse transcribed into cDNA templates, the PCR (3 min at 95°C, followed by 40 amplification cycles of 10 s at 95°C, 10 s at 55°C, and 10 s at 72°C) was performed on the mixed reaction system containing cDNA templates, gene-specific primers (Table 1) and SYBR Green Mix (TOYOBO, Japan). The *β-actin* was used as the reference gene. The relative gene expression was normalized to the control group and calculated by the method of 2^―ΔΔ*C*t^.

**Table 1:** Primers of target genes

Gene	Forward (5′–3′)	Reverse (5′–3′)
*β-actin*	CCGCGAGTACAACCTTCTTG	TGACCCATACCCACCATCAC
*Aggrecan*	ATGGCATTGAGGACAGCGAA	GCTCGGTCAAAGTCCAGTGT
*Collagen II*	GCCAGGATGCCCGAAAATTAG	CCAGCCTTCTCGTCAAATCCT
*p53*	CCTTAAGATCCGTGGGCGT	GCTAGCAGTTTGGGCTTTCC
*p16*	TACCCCGATACAGGTGATGA	TACCGCAAATACCGCACGA

### Western blot analysis

Protein expression of matrix-related molecules (aggrecan and collagen II) and senescence-related molecules (p16 and p53), and activity of the p38 pathway were analyzed by Western blot assay. Briefly, total protein was extracted by RIPA lysis buffer (Beyotime, China) and its concentration was measured by the Protein BCA Kit (Beyotime, China). Then, 60 μg protein in each group was separated by SDS/polyacrylamide gel (SDS/PAGE) and transferred to the PVDF membrane (Beyotime, China). Subsequently, the PVDF membranes were incubated with primary antibodies (β-actin: Abcam, ab8227; p16: Novus, NBP2-37740; p53: Abcam, ab26; aggrecan: Norvus, NB120-11579; collagen II: Abcam, ab185430; p38: Cell Signaling Technology, #8690; p-p38: Cell Signaling Technology, #4511) and horseradish peroxidase (HRP)–conjugated secondary antibodies (Beyotime, China). Finally, the protein bands on the PVDF membrane were visualized by SuperSignal West Pico Trial Kit (Thermo, U.S.A.). The density of each protein band was quantitated using Quantity One Software.

### Statistical analysis

All data were collected from three independent experiments performed in triplicate. Data were presented as mean ± S.D. and analyzed using the SPSS 17.0 software. After homogeneity test for variance, differences between intergroups were analyzed by one-way ANOVA. A *P*-value <0.05 was considered as statistical difference.

## Results

### NP cell proliferation

In the CCK-8 assay (Figure 1A), experimental NP cells had a decreased OD450 value compared with the control NP cells. For the EdU incorporation assay (Figure 1B), the RFU value reflecting EdU incorporation content of the control NP cells was significantly higher than that in the experimental NP cells. However, when the inhibitor SB203580 was added into the experiment NP cells, both OD450 and RFU value were partly increased.

**Figure 1:** Cell proliferation potency of NP cells (**A**) CCK-8 assay. (**B**) EdU incorporation assay. Data are expressed as mean ± S.D. (*n*=3). *: Shows a statistical difference (*P*<0.05) between two groups.

### NP cell cycle analysis

In the cell cycle analysis (Figure 2), we found that experimental NP cells had a significantly increased G_0_/G_1_ phase fraction whereas a decreased S-phase fraction compared with the control NP cells. However, the inhibitor Sb203580 partly reversed the acidic niche’s effects on cell cycle in the experimental NP cells.

**Figure 2:** Cell cycle analysis of NP cells The histogram shows cell fraction proportion of each cell cycle (G_0_/G_1_, S, and G_2_/M).

### Telomerase activity of NP cells

In the telomerase activity analysis (Figure 3), results showed that experimental NP cells had a significantly decreased telomerase activity compared with the control NP cells. Oppositely, the inhibitor SB203580 partly increased telomerase activity in the experimental NP cells.

**Figure 3:** Telomerase activity of NP cells Data are expressed as mean ± S.D. (*n*=3). *: Shows a statistical difference (*P*<0.05) between two groups.

### Expression of senescence-related molecules in NP cells

Real-time PCR analysis showed that mRNA expression of senescence-related markers (p16 and p53) in the experimental NP cells was significantly up-regulated compared with the control NP cells (Figure 4A). Western blot assay also showed that protein expression of p16 and p53 in the experimental NP cells was increased compared with the control NP cells (Figure 4B). Similarly, inhibitor SB203580 partly decreased their expression in experimental NP cells both at gene and protein levels.

**Figure 4:** Analysis of the expression of senescence-related molecules (p16 and p53) in NP cells (**A**) Real-time PCR analysis. (**B**) Western blot analysis. Data are expressed as mean ± S.D. (*n*=3). *: Shows a statistical difference (*P*<0.05) between two groups.

### Expression of matrix-related molecules in NP cells

Gene expression analysis showed that mRNA expression of matrix-related molecules (aggrecan and collagen II) in the experimental NP cells was significantly down-regulated compared with the control NP cells (Figure 5A). Moreover, protein expression of aggrecan and collagen II in the experimental NP cells was decreased compared with the control NP cells (Figure 5B). Additionally, inhibitor SB203580 partly increased their expression in the experimental NP cells both at gene and protein levels.

**Figure 5:** Analysis of the expression of matrix molecules (aggrecan and collagen II) in NP cells (**A**) Real-time PCR analysis. (**B**) Western blot analysis. Data are expressed as mean ± S.D. (*n*=3). *: Shows a statistical difference (*P*<0.05) between two groups.

### Activity of the p38 MAPK pathway

To investigate the role of p38 MAPK pathway in this process, we analyzed expression of p38 MAPK and p-p38 MAPK using Western blot. Results showed that relative expression of p-p38 MAPK (p-p38/p38) in the experimental NP cells was significantly increased compared with the control NP cells. Reasonably, the inhibitor SB203580 significantly inhibited activation of the p38 MAPK pathway (Figure 6).

**Figure 6:** Analysis of activity of the p38 MAPK pathway in NP cells Data are expressed as mean ± S.D. (*n*=3). *: Shows a statistical difference (*P*<0.05) between two groups.

## Discussion

IVD is the largest avascular organ in human body and it degenerates much earlier than other organs in life [22]. Nutrient supply to the disc central NP cells is done mainly through two approaches: the CEP pathway and the peripheral AF pathway [6]. Due to the long diffusion distance of the AF pathway, and the degenerative changes in the CEP, nutrients’ diffusion into the NP region and the metabolism wastes elimination out of the NP region are all restricted [13], which results in a very acidic niche in the disc NP region. Previously, researchers have proved that NP cell senescence is involved in the progression of disc degeneration. However, whether NP cell senescence is associated with the acidic niche of NP region remains unclear. In the present study, we demonstrated for the first time that the acidic pH close to that in a severe degenerative disc significantly promotes NP cell senescence and that activation of the p38 MAPK pathway may be involved in this process.

Due to the structural character, the oxygen tension within the disc central NP region is very low, leading to anaerobic glycolysis of majority NP cells and thus the large amount of lactic acid accumulation [7]. Because the diffusion distance is too long to sufficiently eliminate the lactic acid-like metabolites, the disc NP cells are resided in a very acidic niche *in vivo* [23,24]. According to previous studies, the intradisc pH value ranges from 7.2 in a healthy disc to 6.2 in a severe degenerative disc [12]. There are several studies investigating the effects of acidic environment on disc NP cell biology have reported that a very low acidic niche has detrimental effects on NP cell viability and NP matrix anabolism [8,17,25]. Therefore, the acidic niche may be an important initiator of disc degeneration, and more studies should be done to clearly investigate its detrimental role and mechanism.

Disc degeneration is a complicated process characterized by the age-related alteration and tissue destruction induced by multiple stresses [19]. Cellular senescence is often identified as irreversible growth arrest under various stresses, which is a common approach that mediates age-related dysfunctions and chronic diseases [26,27]. Though cell apoptosis process contributes to a decrease in disc cell number and ECM production [28], cellular senescence has also been identified as an obvious cellular feature within the human and animal degenerative discs [29,30]. Importantly, a positive relationship between disc cell senescence and disc degeneration extent was reported previously [31].

Until now, no studies have reported the effects of acidic niche on NP cell senescence. In the present study, we found that the very acidic pH of 6.2 significantly promoted NP cell senescence compared with the acidic pH of 7.2 close to that in a healthy disc tissue, reflected by the suppressed cell proliferation potency, increased G_0_/G_1_ phase fraction whereas a decreased S-phase fraction, declined telomerase activity and an up-regulated expression of senescence-related molecules (p16 and p53) whereas a down-regulated expression of matrix-related molecules (aggrecan and collagen II) at both gene and protein levels. In-line with us, a previous study has reported that the acidic pH can induce epithelial cellular senescence in reflux esophagitis [20]. The p38 MAPK pathway participates in many cell bioactivities through converting the extracellular stimuli into intracellular responses, such as cell apoptosis, cell proliferation, and cell biosynthesis [32]. In this study, we found that the very acidic pH of 6.2 significantly increased activity of the p38 MAPK pathway compared with the pH of 7.2, and inhibition of the p38 MAPK pathway partly reversed NP cell senescence in the NP cells treated with the acidic pH of 6.2, indicating that the very acidic pH close to that in a severe degenerative disc significantly promotes NP cell senescence through activating the p38 MAPK pathway.

The preent study also has several limitations. First, because the rat disc NP tissue has large amount of notochordal cells, the isolated NP cells in the present study may contain some notochordal cells. This limitation may affect the persuasion of the present study. Second, we just designed a very acidic pH of 6.2 close to that in a severe degenerative disc. A higher acidic pH value close to that in a moderate-degenerative disc may be helpful to observe a dose-dependent effect.

In a word, we studied the effects of different acidic environments on NP cell senescence. Our results demonstrated that the very acidic pH close to that in a severe degenerative disc significantly promotes NP cell senescence through activating the p38 MAPK pathway. The present study will help us to better understand the pathogenesis of disc degeneration, and provides a new mechanism that drives NP cell senescence during disc degeneration.

## Abbreviations

AF: annulus fibrosus
CCK-8: cell counting kit-8
CEP: cartilage endplate
DMEM/F12: Dulbecco’s modified Eagle media:nutrient mixture F-12
ECM: extracellular matrix
IVD: intervertebal disc
LBP: low back pain
NP: nucleus pulposus
PI: propidium iodide
RFU: relative fluorescence unit
